# FOXF1 Was Identified as a Novel Biomarker of Infantile Hemangioma by Weighted Coexpression Network Analysis and Differential Gene Expression Analysis

**DOI:** 10.1155/2022/8981078

**Published:** 2022-07-30

**Authors:** Yuchao Zhang, Ping Wang

**Affiliations:** Department of Vascular Surgery, The Affiliated Huaian No. 1 People's Hospital of Nanjing Medical University, Huaian 223300, China

## Abstract

**Background:**

The most frequent benign tumor in newborns is infantile hemangioma. The majority of infantile hemangiomas has a favorable prognosis and generally fades away on their own. Some people, however, do experience major consequences. Transcriptome alterations in infantile hemangiomas are yet unclear. The use of transcriptome analysis to uncover diagnostic markers for infantile hemangioma has clinical implications.

**Methods:**

The dataset GSE127487 for infantile hemangioma was obtained from the GEO database. The gene set most related with infantile hemangioma was investigated using weighted coexpression network analysis. Differential expression analysis was performed to see whether genes were up or downregulated in infantile hemangiomas. The enrichment of gene sets in pathways or functions is determined via enrichment analysis. Hub genes were discovered via protein-protein interaction network analysis. The relationship between hub genes and immune cells was investigated using immunomicroenvironment analysis.

**Results:**

Turquoise and Pink modules were revealed to be the most linked with infantile hemangioma in a weighted coexpression network analysis (*p* < 0.001). The genes in the two modules were mostly concentrated in actin filament organization, embryonic organ development, reproductive structure development, cell substrate adhesion, extracellular matrix organization, and so on, according to GO enrichment analysis (*p* < 0.05). These gene enrichment pathways comprised the PI3K-Akt signaling pathway, human papillomavirus infection, focal adhesion, and hepatitis C pathways, according to KEGG enrichment analyzes (*p* < 0.05). Differential expressed gene analysis showed 43 upregulated and 21 downregulated genes in infantile hemangiomas. We found the gene set most associated to infantile hemangioma by intersecting the elevated genes with the genes acquired by WGCNA, with FOXF1 serving as the hub gene. FOXF1 was linked to the degree of monocyte infiltration, according to immunocorrelation analysis (*p* < 0.05). B cell memory, dendritic cells resting, macrophage M0, neutrophils, and T cells helper are all negatively connected (*p* < 0.05). In the FOXF1 hyperexpression group, GSEA analysis revealed that cholesterol homeostasis and cell cycle-associated pathways G2M checkpoint were primarily activated (*p* < 0.05).

**Conclusion:**

FOXF1 was found to be a reliable biomarker of infantile hemangiomas in our research of transcriptome changes in infantile hemangiomas.

## 1. Introduction

Infantile hemangioma (IH) is the most frequent tumor in newborns, affecting roughly 5–10% of them [1–3]. IH usually occurs in the first few weeks of life and spreads quickly during childhood [4]. According to the tissue level of growth, IH can be characterized as superficial, deep, or mixed [5]. IH is classified as focal, multifocal, segmental, and so on, depending on the pattern of growth [6]. The perineum, face, limbs, and trunk are common IH locations [7]. Although most IH is benign and has a fair prognosis, there are a number of problems that can have a significant impact on a child's look and quality of life, and extreme complications can even result in death [8]. Therefore, it is critical to stratify the risk of IH patients and look for new biomarkers to help with diagnosis and treatment.

The genomes and transcriptome alterations of IH are yet unclear. Using multiomics approaches to investigate genetic changes in IH can serve as a starting point for the discovery of new IH indicators and the investigation of the immunological microenvironment [9]. In recent years, RNA-sequencing has been utilized to investigate genetic alterations in a variety of disorders. Many biological and medical research studies are increasingly relying on bioinformatics as a result of the rise of bioinformatics [10]. Understanding gene expression regulatory mechanisms is also an important aspect of bioinformatics [11]. The diagnosis and treatment of human diseases are defined in terms of the role of biomolecules in gene regulation. Bioinformatics has emerged as a critical component in the advancement of life science as a whole, as well as the frontier of life science research. GEO is currently one of the most widely used databases in bioinformatics analysis, with gene expression data given by research organizations all over the world, primarily gene chip and high-throughput sequencing data. We used the GEO database to download IH dataset for analysis in this study. Dataset GSE127487, published in 2019, containing 23 IH samples and 5 normal controls, was downloaded for analysis. In the original study, transcriptomic sequencing data were used to reveal potential biomarkers of propranolol for IH: EPAS1, LASP1, SLC25A23, MYO1B, and ALDH1A1. We used this transcriptome data to perform weighted coexpression network analysis and differential expression analysis and identified some new biomarkers for IH [12].

## 2. Methods

### 2.1. Data Download and Processing

The Gene Expression Omnibus (GEO) database (https://www.ncbi.nlm.nih.gov/geo/) is a comprehensive website that collects transcriptome data from a wide range of diseases and clinical data, making it easy for researchers to examine. GSE127487, a dataset encompassing 23 infantile hemangiomas and 5 normal control samples, was retrieved from this database. GPL13607 annotated gene names and averaged several probes belonging to a gene name. The data from the transcriptome were standardized and log2 transformed.

### 2.2. Weighted Coexpression Network Analysis (WGCNA)

Genes with comparable biological roles are classified into clusters in WGCNA analysis, which is based on grouping of gene expression patterns of each sample. The soft threshold range in this study is 0–10 as a continuous integer and 10–20 as an integer with step 2. The pickSoftThreshold function of the function WGCNA package can be used to find the best soft domain value. To execute gene clustering, set the minimum number of module genes to 200 and deepSplit to 2.

### 2.3. Enrichment Analysis of Gene Ontology (GO)

Cellular component (CC), molecular function (MF), and biological process (BP) are the three sections of the GO database. By comparing the given gene list with the gene set of biological functions, the GO database was used to examine the biological functions enriched.

### 2.4. Kyoto Encyclopedia of Genes and Genomes (KEGG) Enrichment Analysis

The gene list provided was matched with genes in human pathways collected by the KEGG database, and the enriched pathway was studied.

### 2.5. Analysis of Differentially Expressed Genes (DEGs)

The “LIMMA” software was used to look for differentially expressed genes in the control and infantile hemangioma groups, with *p* value < 0.05 and | logFC | > 0.5. For visualization, the *R* packages heatmap and ggplot2 are utilized.

### 2.6. Protein-Protein Interaction Network Analysis

STRING<>(https://cn.string-db.org/) is a popular protein interaction analysis website. The site analyzes the organism by inputting a list of genes into a box and selecting *Homo sapiens* as the target species and then downloading and visualizing the results with Cytoscape software. The cytoHubba plug-in was then used to look for other hub genes, which were ordered using the MCC technique.

### 2.7. Immune Cell Infiltration Analysis

The CIBERSORT method is the most widely used method for measuring immune infiltration, and it was utilized to quantify the degree of immune cell infiltration in infantile hemangioma and the control group in this study.

### 2.8. Gene Set Enrichment Analysis (GSEA)

GSEA is a widely used enrichment analysis method that compares genes to a set of genes. GSEA examines if all of the genes in a gene set are clustered at the top or bottom of the multiples of difference list.

## 3. Results

### 3.1. Weighted Coexpression Network Analysis (WGCNA)

WGCNA analysis was performed in this work to look for gene sets that change in conjunction with infantile hemangioma. The best soft domain value found from function computation is 10, as shown in Figure 1(a). The data adhere to the power law distribution when the soft domain value is set to this value, *R*^2^ > 0.8, and when the soft domain value is more than 10, mean connectivity gradually becomes stable. All genes were coclustered into 13 nongray modules, as shown in Figures 1(b) and 1(c), with turquoise and pink being the most closely connected to infantile hemangioma. There was a high positive association between gene significance for body weight and module membership in turquoise and pink modules (COR = 0.92 and *p* < 0.001 and COR = 0.78 and *p* < 0.001), as shown in Figures 1(d) and 1(e). The following analysis comprised genes from the turquoise module, which contains 2,495 genes, and the pink module, which has 673 genes.

### 3.2. GO and KEGG Enrichment Analyses

As shown in Figure 2(a), infantile hemangioma-related genes acquired by WGCNA were primarily enriched in actin filament organization, embryonic organ development, reproductive structure development, cell substrate adhesion, extracellular matrix organization, extracellular structure organization, regulation of small GTPase-mediated signal transduction, positive regulation of ion transport, cell matrix adhesion, cell shape regulation, and so on, as determined by GO enrichment. KEGG enrichment analysis revealed that the PI3K-Akt signaling pathway, human papillomavirus infection, focal adhesion, and hepatitis C were the most enriched, as shown in Figure 2(b).

### 3.3. Differential Expression Gene Analysis and Protein-Protein Interaction Network Construction

By using the differential analysis of limma program, a total of 64 differential genes were screened from infantile hemangioma and the control group, of which 43 were upregulated and 21 were downregulated. The heat map in Figure 3(a) shows differential gene expression in infantile hemangiomas and controls. The volcano map, as shown in Figure 3(b), illustrates the distribution of differential genes, with HSD17B2, IDO1, PCDH12, FCN3, and LIN28B being the most significantly upregulated genes with the lowest *p* value. SERPINA3, SLPI, TC2N, TFF3, and MUC7 were the five genes that were significantly downregulated. 36 genes were determined to be most linked with infantile hemangioma when the turquoise and pink modules were intersected with these upregulated genes. The interaction between these proteins is shown in Figure 3(c). FOXF1 was identified as the top hub gene by the CytoHubba plug-in.

### 3.4. Expression and Diagnostic Value of FOXF1 in Infantile Hemangioma

FOXF1 was found to be strongly expressed in infantile hemangiomas (*p* < 0.001), as shown in Figure 4(a). ROC and PRC analyses were used to further investigate the diagnostic significance of this gene in infantile hemangioma. The AUC of ROC analysis was 0.97, while the AUC of PRC analysis was 0.99, indicating that FOXF1 is a reliable marker for the diagnosis of infantile hemangioma, as shown in Figure 4(b).

### 3.5. Immune Cell Infiltration Analysis

The CIBORSORT algorithm was used to assess the degree of immune cell infiltration in infantile hemangiomas. Mast cells make up a significant fraction, as shown in Figure 5(a). Mast cells resting identified higher infiltration in the FOXF1 high expression group, as shown in Figure 5(b). Whereas, macrophages M0 had a lower degree of infiltration (*p* < 0.05). FOXF1 is favorably connected with monocyte infiltration degree, whereas it is negatively correlated with B cell memory, dendritic cells resting, macrophage M0, neutrophils, and T cells follicular helper (*p* < 0.05), according to correlation analysis (Figures 5(c)–5(h)).

### 3.6. GSEA Analysis

The cholesterol homeostasis and cell cycle-associated pathways G2M CHECKPOINT were primarily activated in the FOXF1 hyperexpression group, as shown in Figures 6(a) and 6(b).

## 4. Discussion

The most common benign tumor in children, infantile hemangioma (IH), has a distinct development pattern [13]. IH grows rapidly before the age of eight weeks and is essentially mature before the age of five months, with the majority of spontaneous regression [13]. For the treatment of early IH, beta-blockers are suggested [14]. However, beta-blockers have limited clinical efficacy in some patients [14]. Furthermore, some children (approximately 10%) still suffer evident clinical consequences, such as blindness, ulceration, infection, and even heart failure, which cause many children's lives to be ruined and even harm them for the rest of their lives [15]. As a result, early and reliable biomarkers for IH are needed to guide IH diagnosis and treatment.

Bioinformatics analysis was employed to investigate transcriptome changes in IH in depth in this work. To begin, weighted coexpression network analysis (WGCNA) was utilized to look at the modules that were most closely linked to IH. Turquoise and pink modules were found to have a strong correlation with IH. Then, we did an enrichment analysis of those genes and discovered that they were mostly involved in actin filament organization, embryonic organ development, reproductive structure development, cell substrate adhesion, extracellular matrix organization, extracellular structure organization, regulation of small GTPase mediated signal transduction, positive regulation of ion transport, cell matrix adhesion, cell shape regulation, and so on. The PI3K-Akt signaling pathway, human papillomavirus infection, focal adhesion, and hepatitis C, among others, are heavily represented in the pathways of these genes. This provides insights into the mechanisms of these genes and their interactions in infantile hemangiomas. FOXF1 was identified as a critical gene for IH after further protein-protein interaction network research. FOXF1 was considerably upregulated in IH, according to expression analysis, and the ROC curve revealed that FOXF1 had a very high AUC value and good diagnostic accuracy. FOXF1 was shown to be connected with various immune cells in IH, most of which were negatively correlated, but favorably correlated with monocytes, according to a subsequent investigation of the immunological microenvironment. This serves as a starting point for learning more about FOXF1's significance in the immunological background of IH. Finally, gene set enrichment analysis (GSEA) revealed significant cholesterol homeostasis and G2M checkpoint pathway enrichment in the FOXF1 high expression group.

FOXF1 belongs to the forkhead-box (FOX) family of proteins and is involved in cell proliferation, differentiation, embryogenesis, and longevity [16–18]. The FOX family is also involved in transcription and DNA repair control. The importance of FOXF1 in many human diseases has been preliminarily elucidated, particularly in various malignancies, at this time. Milewski et al. found that FOXF1 is downstream of PAX3-FOXO1 in rhabdomyosarcoma, promoting tumor development, and FOXF1 may be a potential therapeutic target for rhabdomyosarcoma [19]. Zhao et al. discovered that epigenetic activation of FOXF1 allows cisplatin-resistant NSCLC to acquire stem cell characteristics [20]. FOXF1 increases tumor spread in colorectal cancer by activating SNAI1 and causing epithelial-mesenchymal transition (EMT), according to Wang et al. [21]. Not only that, FOXF1 has also been shown to play an important role in benign disease. FOXF1 knockdown enhances Wnt/*β*-catecholamine activation, which enables bone marrow-derived mesenchymal stem cell osteogenesis and protects bone loss after oophorectomy, according to Shen et al. [22]. Sturtzel et al. discovered that FOXF1 is involved in the germination of endothelial progenitor cells and linked blood vessels, which may be implicated in tissue neovascularization [23]. Our study reveals the value of FOXF1 in infantile hemangiomas, where the role of FOXF1 was previously unknown. FOXF1 has a high AUC value in infantile hemangioma, and the AUC value in both ROC curve and PRC curve is greater than 0.9, indicating that FOXF1 is very robust in the diagnosis of infantile hemangioma. FOXF1 has also been linked to a number of immune cells, shedding light on the pathophysiology of infantile hemangiomas and the intricate interaction that occurs.

## 5. Conclusion

In conclusion, our research looked at transcriptome changes in infantile hemangioma and found FOXF1 to be a novel biomarker of infantile hemangioma with a good diagnostic value using several analysis approaches. Our research, however, has certain limitations. We do not have enough relevant in vitro and in vivo studies to verify FOXF1's influence, but that will change in the future.

## Figures and Tables

**Figure 1:** Weighted coexpression network analysis (WGCNA). (a) The best soft domain value found from function computation is 10. (b)-(c) All genes coclustered into 13 nongray modules with turquoise and pink being the most closely connected to infantile hemangioma. (d)-(e) Association between gene significance for body weight and module membership in turquoise and pink modules (COR = 0.92 and *p* < 0.001 and COR = 0.78 and *p* < 0.001).

**Figure 2:** (a) GO and (b) KEGG enrichment analyses.

**Figure 3:** Differential expression gene analysis and protein-protein interaction network construction. (a) The heat map of differential gene expression in infantile hemangiomas and controls. (b) The volcano map. (c) The interaction between these proteins. FOXF1 was identified as the top hub gene by the CytoHubba plug-in.

**Figure 4:** Expression and diagnostic value of FOXF1 in infantile hemangioma. (a) FOXF1 found to be strongly expressed in infantile hemangiomas (*p* < 0.001). (b) The AUC of ROC analysis is 0.97 and PRC analysis is 0.99.

**Figure 5:** Immune cell infiltration analysis. (a) The degree of immune cell infiltration in infantile hemangiomas. (b) Mast cells resting identified higher infiltration in the FOXF1 high expression group. Whereas, macrophages M0 had a lower degree of infiltration (*p* < 0.05). (c)–(h) Immune correlation analysis.

**Figure 6:** (a)-(b) GSEA analysis.

## Data Availability

The data used to support the findings of this study are included within the article.
